The article "Research Value of Intensity Modulated Radiation Therapy in Alleviating Parotid Gland Function Injury in Patients with Stage N0 Nasopharyngeal Carcinoma from Physical and Dosimetric Aspects" was retracted in 2023. Reasons: unreliable results or conclusions; lack of ethics approval or compliance; concerns about the data; concerns about the results or conclusions.

# Research Value of Intensity Modulated Radiation Therapy in Alleviating Parotid Gland Function Injury in Patients with Stage N0 Nasopharyngeal Carcinoma from Physical and Dosimetric Aspects

**DOI:** 10.1155/2022/4651364

**Published:** 2022-07-11

**Authors:** Lirong Zheng, Hong Wang, Neng Yang, Fenglei Du, Lin Xiao, Gangfeng Wu

**Affiliations:** ^1^Department of E.N.T, Taizhou Hospital of Zhejiang Province Affiliated to Wenzhou Medical University, Taizhou, 317000 Zhejiang, China; ^2^Department of Pharmacy, Taizhou Hospital of Zhejiang Province Affiliated to Wenzhou Medical University, Taizhou, 317000 Zhejiang, China; ^3^Department of Radiotherapy, Cancer Hospital of the University of Chinese Academy of Sciences (Zhejiang Cancer Hospital), Hangzhou, 310000 Zhejiang, China; ^4^Department of Otolaryngology, Taizhou Enze Medical Center (Group) Enze Hospital, Taizhou, 317000 Zhejiang, China; ^5^Department of E.N.T, Taizhou Second People's Hospital, Taizhou, 317000 Zhejiang, China

## Abstract

**Objective:**

To study the feasibility of intensity modulated radiation therapy (IMRT) for stage N_0_ nasopharyngeal carcinoma (NPC) and its parotid gland (PG) function preservation from physical and dosimetric aspects.

**Methods:**

All the clinical data of 77 patients with pathologically confirmed T_1-4_N_0_M_0_ NPC who received radiotherapy between July 2017 and October 2019 in the Radiotherapy Center of Taizhou Hospital of Zhejiang Province affiliated to Wenzhou Medical University were analyzed retrospectively. Three-dimensional conformal radiotherapy (3D-CRT) and IMRT were used in 35 and 42 cases, respectively. The treatment efficiency and the dosimetry differences of the PG in the intensity modulation plan were compared between groups. Quantitative monitoring of 99mTc radionuclide imaging of PG was performed before, at the end of, and 3, 6, and 12 months after radiotherapy. The degree of PG function injury and xerostomia was compared between groups at the end of radiotherapy and 12 months later.

**Results:**

Higher minimal, maximal, and average irradiation doses of PG were determined in 3D-CRT-treated patients compared with IMRT-treated cases (*P* < 0.05). Compared with before radiotherapy, the PG uptake index (UI) and excretion index (EI) of both cohorts of patients decreased to varying degrees at the end of radiotherapy, with PG function injury and xerostomia symptoms observed in all cases but with no obvious difference between groups (*P* > 0.05). To a certain extent, the PG function recovered and the xerostomia symptoms relieved in both groups 12 months after radiotherapy, with better improvements in IMRT group versus 3D-CRT group.

**Conclusion:**

IMRT has similar short-term efficacy to 3D-CRT in treating patients with stage N_0_ NPC, but it can effectively reduce the dose of PG radiotherapy and protect the PG function on the premise of ensuring sufficient tumor coverage and dose, showing certain dosimetry advantages.

The article "Research Value of Intensity Modulated Radiation Therapy in Alleviating Parotid Gland Function Injury in Patients with Stage N0 Nasopharyngeal Carcinoma from Physical and Dosimetric Aspects" was retracted in 2023. Reasons: unreliable results or conclusions; lack of ethics approval or compliance; concerns about the data; concerns about the results or conclusions.

## 1. Introduction

As a malignancy occurring at the top and lateral wall of the nasopharyngeal cavity, nasopharyngeal carcinoma (NPC) inflicts 133,000 new cases in 2020, accounting for 0.7% of all cancers worldwide [1]. NPC is unsuitable for surgical treatment due to its unique biological characteristics, pathological types, and physiological anatomical location [2–4]. Radiotherapy is currently the preferred clinical treatment for NPC in clinic [5]. Meanwhile, concurrent chemoradiotherapy may be combined with neoadjuvant chemotherapy, which is also the best choice for locally advanced (stage II-IVa) NPC [6, 7]. With the upgrading of radiotherapy equipment and the rapid development of engineering physics and imaging technology, radiotherapy has gone through several stages: conventional 2-dimensional radiotherapy (2D-RT) [8], 3-dimensional conformal radiotherapy (3D-CRT) [9], and intensity modulated radiation therapy (IMRT) [10]. 3D treatment planning makes it possible to better visualize the anatomy and improve target delineation, thus avoiding doses to normal structures. However, since each of the 3-4 beams used for treatment lacks dose regulation, a large amount of dose is still delivered to normal tissue [11]. At present, IMRT is the mainstream radiotherapy method in treating NPC. IMRT technology adjusts the dose distribution in the radiation field in all directions according to the needs of the objective function, so as to better match the high-dose region to the target area in the three-dimensional direction and lower the radiation dose to the adjacent normal counterparts [12, 13]. IMRT costs more and requires more logistics from the start of treatment planning through the physical quality assurance process. A retrospective comparative study showed that the dose advantage of IMRT over 3D-CRT improved patients' clinical outcomes [14].

Parotid gland (PG), as one of the glands excreting saliva [14], plays a vital part in protecting oral health. Today, the survival time of patients has been prolonged as the treatment technology improves, accompanied by some after-effects brought by relevant treatment, resulting in an increasing attention in patients' quality of life (QOL) [15]. Among them, PG, which is highly sensitive to radiotherapy, will inevitably receive a certain dose of radiation due to the limitation of radiotherapy technology and limited target area [16]. It is well known that even 10-15 Gy can affect the PG in traditional fractionated radiotherapy. Although the PG function may recover with time after 40-50 Gy irradiation, large-dose irradiation can cause irreversible damage to the PG function, seriously damaging the patient's taste, language, and other related functions [17, 18]. This kind of injury will not threaten the patient's life, but will seriously compromise the patient's QOL. Now, IMRT is gaining popularity in the treatment of NPC, due to findings that suggest a significant incremental improvement in dose distribution in a three-dimensional conformal plan, encouraging local control and protection of PG function [19]. Hence, it is of great clinical implications to explore a therapeutic strategy for minimizing PG disorders in NPC cases treated with radiotherapy. Related studies have shown that IMRT can significantly lower the radiation dose of PG, reduce subsequent adverse events, and restore the patient's secretory function [20].

The article "Research Value of Intensity Modulated Radiation Therapy in Alleviating Parotid Gland Function Injury in Patients with Stage N0 Nasopharyngeal Carcinoma from Physical and Dosimetric Aspects" was retracted in 2023. Reasons: unreliable results or conclusions; lack of ethics approval or compliance; concerns about the data; concerns about the results or conclusions.

Therefore, how to reduce the irradiation dose and volume of PG irradiated while ensuring the treatment volume of the target area, so as to preserve the PG function, reduce the incidence and severity of xerostomia (XS) symptoms, and improve the QOL of patients, has become a problem to be solved in radiotherapy for NPC. The novelty and motivation of this work lie in clarifying the protective action of IMRT against parotid dysfunction in stage N_0_ NPC patients from the dosimetric point of view, which hopefully provide scientific basis for optimizing the dose in neck clinical target area of nasopharyngeal carcinoma.

## 2. Data and Methods

### 2.1. Study Population

All the clinical data of 77 pathologically confirmed T_1-4_N_0_M_0_ NPC patients who received radiotherapy between July 2017 and October 2019 in the Radiotherapy Center of Taizhou Hospital of Zhejiang Province affiliated to Wenzhou Medical University were analyzed retrospectively. Among them, 35 patients were treated with 3D-CRT, including 19 males and 16 females aged 23-71 years (median age: 45); T1, T2, T3, and T4N_0_M_0_ NPC were found in 4, 11, 3, and 17 cases, respectively. 42 patients were treated with IMRT, including 24 males and 18 females aged 20-69 years (mean: 46). In terms of clinical staging, 6 cases were in stage T1, 12 in stage T2, 6 in stage T3, and 18 in stage T4. Inclusion criteria: (1) no history of PG-related diseases, (2) the Eastern Cooperative Oncology Group (ECOG) grading [21] ≤1, (3) Karnofsky performance scale (KPS) score [22] ≥80, (4) follow-up time > 12 months, and (5) complete clinical data. Exclusion criteria: (1) abnormal hepatorenal, cardiac, or pulmonary function; (2) other serious systemic diseases; and (3) incomplete clinical data. No statistical differences were observed in general data between groups, which were comparable (*P* > 0.05). This research was carried out after obtaining approval from the Medical Ethics Committee of Taizhou Hospital of Zhejiang Province affiliated to Wenzhou Medical University.

The article "Research Value of Intensity Modulated Radiation Therapy in Alleviating Parotid Gland Function Injury in Patients with Stage N0 Nasopharyngeal Carcinoma from Physical and Dosimetric Aspects" was retracted in 2023. Reasons: unreliable results or conclusions; lack of ethics approval or compliance; concerns about the data; concerns about the results or conclusions.

### 2.2. Treatment Methods

All patients were placed in a comfortable supine position, so as to make a U-shaped thermoplastic mask for their heads. CT scanning was performed after fixing the patient's posture with the headframe and thermoplastic mask, covering the whole skull, nasopharynx, oropharynx, and the whole neck, with a layer spacing of 3 mm. After the scan, CT images were transmitted to the Eclipse planning system (TPS) to outline vital organs for reconstruction, planning, calculation, and evaluation. According to enhanced CT and MRI images and by referring to ICRU reports nos. 50 and 62, the radiotherapy target area marked, which composed of clinical target volume (CTV), gross tumor volume (GTV), and planning target volume (PTV), was delineated layer by layer by physicians. PTV was automatically generated by TPS according to uncertain factors, which were PGTVnx, PTV1, and PTV2, respectively. The related organs at risk (OARs) like spinal cord, brainstem, temporal lobe, eyeball, optic nerve, PG, and temporomandibular joint were sketched, so that the dose of specific OAR was within the corresponding dose limit [23]. The planning organ at risk volume (PRV) referred to the areas that extend 3 mm from the OAR. In IMRT group, an iX linear accelerator made by VARIAN Inc. of USA was used, and the radiation energy was 6 MV. The prescription doses of PGTVnx, PTV1, and PTV2 were 68 Gy/30 times, 60 Gy/30 times, and 54 Gy/30 times, respectively, 5 times per week. The dose of shrinkage field in 3D-CRT group was increased when irradiated for 20 times, so that the dose of the primary tumor reached the radical dosage.

### 2.3. Endpoints

1. *Clinical Effect Evaluation*. The short-term efficacy of all patients after radiotherapy was evaluated by referring to the World Health Organization (WHO) Response Evaluation Criteria In Solid Tumors [24]. Complete response (CR) referred to disappearance of all lesions; partial response (PR) was indicated if symptoms were obviously relieved, and the lesion volume was reduced by 30-50% compared with the pretreatment value; stable disease (SD) referred to no obvious improvement in symptoms nor decrease in lesion volume; progressive disease (PD) was considered if symptoms deteriorated further, and even new lesions appeared. Response rate = (RG + PR) cases/total cases × 100%
2. *Evaluation of PG Function Injury*. The PG imaging instrument used was DISCOVERY VH of GE Inc. in the United States. The imaging agent 99mTcO4 was freshly leached by a 99Mo-99mTc generator and was intravenously injected with a dose of 370Mb1q. The image was dynamically and continuously collected for 30 min. At the 20th minute, 200 mg Vit C was administered sublingual to patients, and then, the images were collected dynamically for 10 min. The region of interest (ROI) of salivary glands was delineated by the region-of-interest technique, and the excretion index (EI) and uptake index (UI) following acid stimulation were counted by software based on the radioactivity count of skull. The changes of parotid uptake and excretion function before, at the end of, and 3, 6, and 12 months after radiotherapy were analyzed. EI = (apparent diffusion coefficient (ADC) value at acid stimulation − ADC value at 6 min after acid stimulation)/(ADC value on acid stimulation − base value); UI = (peak − base)/base [25]
3. *PG Function Injury Grading [* 26 *]*. Grade I: no obvious injury, with intake and excretion function decline < 20%; grade II: mild impairment, with 20% < uptake and excretion function decline ≤ 40%; grade III: moderate impairment, with 40% < uptake and excretion function decline ≤ 60%; grade IV: severe injury, with 60% < uptake and excretion function decline ≤ 80%; grade V: extreme injury, with uptake and excretion function decline > 80%
4. Degree of Xerostomia. The degree of xerostomia was assessed according to the RTOG/EORTC acute radiation morbidity grading criteria [27]. Grade 0: no change nor obvious XS; grade 1: presence of mild XS, sticky saliva, and changes in taste, all of which caused no changes in eating; grade 2: obvious XS, together with thickening and sticky saliva, and obvious changes in taste; grade 3: severe XS that not allowed for eating dry food, and liquid input was required for maintenance

The article "Research Value of Intensity Modulated Radiation Therapy in Alleviating Parotid Gland Function Injury in Patients with Stage N0 Nasopharyngeal Carcinoma from Physical and Dosimetric Aspects" was retracted in 2023. Reasons: unreliable results or conclusions; lack of ethics approval or compliance; concerns about the data; concerns about the results or conclusions.

### 2.4. Statistical Processing

SPSS 20.0 statistical software (IBM, New York, USA) was used for statistical analysis. The intergroup differences of normally distributed quantitative data represented by mean ± standard deviation were identified by an independent sample *t*-test. A Chi-square test was adopted to test counting data represented by *n* (%). Differences were markedly significant when *P* < 0.05.

## 3. Results

### 3.1. Clinical Efficacy of the Two Groups

The clinical response rate in 3D-CRT and IMRT groups was 77.1% and 85.7%, respectively, showing no statistical difference (*χ*^2^ = 0.0960, *P* = 0.7566) Table 1.

### 3.2. PG Irradiation Doses of Two Radiotherapy Methods

While giving sufficient irradiation dosage to the target area, the irradiation dose to normal counterparts should be controlled within the required limited dose, so as to ensure the effectiveness and safety of treatment. Comparing the minimal, maximal, and average irradiation volumes of the two radiotherapy methods and the doses received by 20%, 30%, and 40% of the PG, it was found that the PG irradiation doses of 3D-CRT-treated patients were significantly higher than those in cases treated with IMRT, and the difference was statistically significant (*P* < 0.05) Table 2.

### 3.3. Parotid Function Imaging before and after Radiotherapy in Two Groups

At the end of radiotherapy and a period after radiotherapy, the UI and EI of PG dropped in both cohorts compared with the preradiotherapy values. However, patients treated with IMRT showed lower UI from 6 months after radiotherapy and lower EI from 3 months after radiotherapy than 3D-CRT treated cases (*P* < 0.05) Table 3.

### 3.4. Functional Impairment of PG in Two Groups

After radiotherapy, 4 cases in the 3D-CRT group developed grade IV PG functional impairment, versus 2 cases in the IMRT group. Patients in the two cohorts showed no evident difference in PG function at the end of radiotherapy (*P* > 0.05). Twelve months later, the PG function recovered in both 3D-CRT and IMRT groups and was better in the IMRT group (*P* < 0.05) Table 4.

### 3.5. Grading of XS in Two Groups

No patients developed grade 3 XS at the end of and 12 months after radiotherapy. The number of cases with grade 1 and grade 2 XS at the end of radiotherapy in 3D-CRT group was 13 and 22, respectively, while that in IMRT group was 18 and 24, respectively, without any significance between groups (*P* > 0.05). Improvement in XS was observed 12 months later in both cohorts, with 10 cases of grade 0, 10 cases of grade 1, and 15 cases of grade 2 in 3D-CRT group, while 16 cases of grade 0, 19 cases of grade 1, and 7 cases of grade 2 in IMRT group, showing statistical significance between groups (*P* < 0.05) Table 5.

## 4. Discussion

Clinically, radiotherapy, with the target site radiation dose directly associated with the local tumor control rate, is the preferred treatment for NPC [28]. During radiotherapy for NPC patients, the PG is inevitably exposed to a certain dose of radiation, which results in XS symptoms that affect the patient's chewing, swallowing, and taste functions. Dry and ruptured oral mucosa will also cause pain, interfere with the patient's sleep, and even lead to oral infection and radioactive dental caries, seriously affecting the patient's QOL and treatment compliance [29, 30]. Although the mechanism of radiation-induced PG volume reduction has not been clarified, it has been reported that it may be due to acinar cell loss or fibrosis, while the recovery of PG volume may be attributed to acinar cell regeneration [31, 32]. Therefore, PG function preservation has become a goal in the treatment of NPC patients.

The article "Research Value of Intensity Modulated Radiation Therapy in Alleviating Parotid Gland Function Injury in Patients with Stage N0 Nasopharyngeal Carcinoma from Physical and Dosimetric Aspects" was retracted in 2023. Reasons: unreliable results or conclusions; lack of ethics approval or compliance; concerns about the data; concerns about the results or conclusions.

This study compared the treatment outcome and radiation dose of N_0_ NPC patients with either 3D-CRT or IMRT. The results showed that the minimum (13.4 ± 2.3 Gy), maximum (56.8 ± 4.3 Gy), and average (31.2 ± 3.3 Gy) radiation dosages of PG in patients with 3D-CRT treatment were significantly higher compared with those receiving IMRT (minimum: 6.6 ± 1.5 Gy; maximum: 50.3 ± 3.7 Gy; average: 24.5 ± 2.8 Gy). To a certain extent, PG function recovered and XS symptoms relieved in both cohorts at 12 months after radiotherapy, with better improvements in IMRT group. Eisbruch et al. [33, 34] studied the dose-volume relationship of PG and found that the PG function of patients could be well preserved if the mean radiation dose of PG was under 24 Gy under nonstimulated conditions or less than 26 Gy under stimulated conditions, that is, under nonstimulated conditions, the salivary secretion can be restored to 76% of the preirradiation on average, and the PG secretion can be restored to 114% of the preirradiation on average under stimulated conditions. However, once the threshold dose is exceeded, parotid function will be difficult to recover. Blanco et al. [35] analyzed head and neck cancer (HNC) patients who received 3D-CRT or IMRT. The authors found that the secretion of unilateral PG decreased after irradiation, and the rate of decline was 5% of the average dose of 1 Gy. When the irradiated dose to the PG reached 25.8 Gy, the salivary flow of a single PG decreased to 25% of its pretreatment value, and the average stimulated parotid salivary (SPS) flow recovered 6 to 12 months after radiotherapy. The results showed that the dose-volume relationship was closely related to the SPS flow of the PG, and the incidence of xerostomia symptoms decreased significantly when the average dose was <25.8 Gy to the PG. Xerostomia, a common complication of HNC after radiotherapy, affects 60-90% of patients, especially their long-term well-being [36]. With the continuous increase of radiation-induced toxicity, it is often aggravated by the simultaneous use of systemic therapy, which has prompted the de intensification of radiotherapy dose in a specific HNC patient cohort [37, 38]. Previous studies also showed that without compromising treatment efficacy, IMRT lowered the incidence of xerostomia by limiting irradiation dose to the salivary glands, which is consisted with our results [39, 40].

The pathological changes of radiotherapy-induced PG function injury are mainly acute inflammatory reactions of PG caused by radiation. In the later stage of injury, there will be gland atrophy, compensatory hyperplasia of adipocytes, central necrosis of glandular lobules and PG related blood vessels, lymphatics, and nerves necrosis, resulting in impaired saliva secretion and excretion function [41]. Salivary gland scintigraphy (SGS) is to evaluate salivary gland function through the ability of salivary gland to absorb and excrete radionuclides. Compared with salivary gland flow measurement, SGS is noninvasive, accurate, and reproducible, so it is widely used in salivary gland function evaluation [5]. Pertechnetate 99mTc is the commonly used radionuclide in salivary gland imaging to measure PG UI and salivary EI after acid stimulation for a certain period of time, thus quantitatively evaluating salivary gland uptake and excretion function [42]. Our study revealed that the UI and EI of PG in both groups decreased at the end of radiotherapy and a period after radiotherapy compared with the preradiotherapy values. In addition, the UI of patients treated with IMRT showed lower UI from 6 months after radiotherapy and EI from 3 months after radiotherapy compared with 3D-CRT-treated cases. Raza et al. [43] used PG imaging to monitor the PG function in 50 cases of thyroid cancer treated with high dose I131, which also demonstrated the feasibility of PG imaging in monitoring PG function injury.

The article "Research Value of Intensity Modulated Radiation Therapy in Alleviating Parotid Gland Function Injury in Patients with Stage N0 Nasopharyngeal Carcinoma from Physical and Dosimetric Aspects" was retracted in 2023. Reasons: unreliable results or conclusions; lack of ethics approval or compliance; concerns about the data; concerns about the results or conclusions.

However, this study still has room for improvement. Due to the limited time frame, the small number of enrolled patients, and the absence of follow-up regarding patients' long-term survival, the research results may be affected to a certain extent. Meanwhile, optimization of clinical target delineation is equally important. Besides, instead of collecting more relevant diagnosis and treatment data from other hospitals, we only studied NPC patients in one hospital with insufficient case data, which may result in some deviation. Thus, in further studies, a large sample size and multicenter survey is needed to obtain more detailed and objective data.

## 5. Conclusion

To sum up, from the dosimetric point of view, IMRT technology for N_0_ NPC can effectively reduce the radiotherapy dose of PG on the premise of ensuring sufficient tumor coverage and dose, which is worth further exploring in clinic.

## Figures and Tables

**Table 1:** Clinical efficacy comparison.

Groups	Complete response	Partial response	Stable disease	Progressive disease	Total effective rate
3D-CRT group (*n* = 35)	20 (57.1)	7 (20.0)	4 (11.4)	4 (11.4)	27 (77.1)
IMRT group (*n* = 42)	25 (59.5)	11 (26.2)	4 (9.5)	2 (4.8)	36 (85.7)
*χ* ^2^					0.0960
*P*					0.7566

**Table 2:** Parotid gland radiation dose of two groups of patients.

Parotid irradiation dose	3D-CRT group (*n* = 35)	IMRT group (*n* = 42)	*t*	*P*
Average irradiation dose (Dmean, Gy)	31.2 ± 3.3	24.5 ± 2.8	9.6396	<0.0001
Maximum irradiation dose (Dmax, Gy)	56.8 ± 4.3	50.3 ± 3.7	7.1301	<0.0001
Minimum irradiation dose (Dmin, Gy)	13.4 ± 2.3	6.6 ± 1.5	15.5984	<0.0001
V20%	59.8 ± 8.6	49.2 ± 10.1	4.9013	<0.0001
V30%	47.8 ± 9.6	33.8 ± 7.2	7.3051	<0.0001
V40%	34.8 ± 9.8	22.4 ± 6.7	6.5665	<0.0001

Notes: Dmean: mean dose; Dmin: minimum dose; Dmax: maximum dose.

The article "Research Value of Intensity Modulated Radiation Therapy in Alleviating Parotid Gland Function Injury in Patients with Stage N0 Nasopharyngeal Carcinoma from Physical and Dosimetric Aspects" was retracted in 2023. Reasons: unreliable results or conclusions; lack of ethics approval or compliance; concerns about the data; concerns about the results or conclusions.

**Table 3:** Comparison of quantitative determination results of 99mTc radionuclide imaging of the parotid gland before and after radiotherapy between the two groups.

	3D-CRT group (*n* = 35)	IMRT group (*n* = 42)	*t*	*P*
Before radiotherapy				
UI	6.26 ± 0.73	6.33 ± 0.74	0.4159	0.6787
EI	0.67 ± 0.36	0.72 ± 0.33	0.6352	0.5272
At the end of radiotherapy				
UI	5.59 ± 0.63	5.40 ± 0.60	1.3526	0.1803
EI	0.59 ± 0.31	0.50 ± 0.35	1.1828	0.2406
3 months after radiotherapy				
UI	4.75 ± 0.70	4.67 ± 0.66	0.5152	0.6079
EI	0.49 ± 0.19	0.41 ± 0.15	2.0646	0.0424
6 months after radiotherapy				
UI	4.76 ± 0.57	4.18 ± 0.45	4.9893	<0.0001
EI	0.52 ± 0.21	0.34 ± 0.18	4.0503	0.0001
12 months after radiotherapy				
UI	5.07 ± 0.46	4.10 ± 0.38	10.1353	<0.0001
EI	0.55 ± 0.36	0.33 ± 0.23	3.2465	0.0017

Notes: UI: uptake index; EI: excretion index.

**Table 4:** Comparison of parotid gland function injury after radiotherapy.

Classification	At the end of radiotherapy		12 months after radiotherapy	
	3D-CRT (*n* = 35)	IMRT (*n* = 42)	3D-CRT (*n* = 35)	IMRT (*n* = 42)
I	18 (51.4)	30 (71.4)	25 (71.4)	39 (92.9)
II	8 (22.9)	5 (11.9)	8 (22.9)	2 (4.8)
III	5 (14.3)	5 (11.9)	2 (5.7)	1 (2.4)
IV	4 (11.4)	2 (4.8)	0 (0.0)	0 (0.0)
V	0 (0.0)	0 (0.0)	0 (0.0)	0 (0.0)
*χ* ^2^	3.7543		6.4122	
P	0.2893		0.0405	

**Table 5:** Comparison of xerostomia grading after radiotherapy.

Classification	At the end of radiotherapy		12 months after radiotherapy	
	3D-CRT group (*n* = 35)	IMRT group (*n* = 42)	3D-CRT group (*n* = 35)	IMRT group (*n* = 42)
0	0 (0.0)	0 (0.0)	10 (28.6)	16 (38.1)
1	13 (37.1)	18 (42.9)	10 (28.6)	19 (45.2)
2	22 (62.9)	24 (57.1)	15 (42.9)	7 (16.7)
3	0 (0.0)	0 (0.0)	0 (0.0)	0 (0.0)
*χ* ^2^	0.2592		6.4262	
P	0.6107		0.0402	

## Data Availability

The labeled dataset used to support the findings of this study are available from the corresponding author upon request.
